# Susceptibility to Infection and Immune Response in Insular and Continental Populations of Egyptian Vulture: Implications for Conservation

**DOI:** 10.1371/journal.pone.0006333

**Published:** 2009-07-22

**Authors:** Laura Gangoso, Juan M. Grande, Jesús A. Lemus, Guillermo Blanco, Javier Grande, José A. Donázar

**Affiliations:** 1 Department of Conservation Biology, Estación Biológica de Doñana (CSIC), Sevilla, Spain; 2 Department of Ecology and Evolution, University of Lausanne, Biophore, Lausanne, Switzerland; 3 Department of Biology, University of Saskatchewan, Saskatoon, Saskatchewan, Canada; 4 Department of Evolutionary Ecology, Museo de Ciencias Naturales (CSIC), Madrid, Spain; University of California, Berkeley, United States of America

## Abstract

**Background:**

A generalized decline in populations of Old World avian scavengers is occurring on a global scale. The main cause of the observed crisis in continental populations of these birds should be looked for in the interaction between two factors - changes in livestock management, including the increased use of pharmaceutical products, and disease. Insular vertebrates seem to be especially susceptible to diseases induced by the arrival of exotic pathogens, a process often favored by human activities, and sedentary and highly dense insular scavengers populations may be thus especially exposed to infection by such pathogens. Here, we compare pathogen prevalence and immune response in insular and continental populations of the globally endangered Egyptian vulture under similar livestock management scenarios, but with different ecological and evolutionary perspectives.

**Methods/Principal Findings:**

Adult, immature, and fledgling vultures from the Canary Islands and the Iberian Peninsula were sampled to determine a) the prevalence of seven pathogen taxa and b) their immunocompetence, as measured by monitoring techniques (white blood cells counts and immunoglobulins). In the Canarian population, pathogen prevalence was higher and, in addition, an association among pathogens was apparent, contrary to the situation detected in continental populations. Despite that, insular fledglings showed lower leukocyte profiles than continental birds and Canarian fledglings infected by *Chlamydophila psittaci* showed poorer cellular immune response.

**Conclusions/Significance:**

A combination of environmental and ecological factors may contribute to explain the high susceptibility to infection found in insular vultures. The scenario described here may be similar in other insular systems where populations of carrion-eaters are in strong decline and are seriously threatened. Higher susceptibility to infection may be a further factor contributing decisively to the extinction of island scavengers in the present context of global change and increasing numbers of emerging infectious diseases.

## Introduction

Recent research has revealed the worrying conservation status of Palearctic avian scavenger populations [1]–[3]. Besides well-documented threats such as habitat degradation, the decline of wild prey populations and human persecution, the relevance of the combination of two additional factors - changes in livestock managing including the regular use of veterinary drugs, and disease - has recently become apparent [1], [4]–[6]. The increased stabling of livestock together with the ban on abandoning carcasses in the field has severely reduced food availability in the countryside [7], and at the same time, the food now available for vultures increasingly consists of intensively raised livestock that is regularly treated with veterinary drugs (mainly antibiotics)[5]. The direct or indirect ingestion of harmful chemical residues from these drugs may pass on to and directly kill scavengers (e.g. the anti-inflammatory drug diclofenac causes renal failure in *Gyps bengalensis* and is thought to be responsible of the crash of several vultures populations all across the Indian subcontinent [1], [4]). In other cases, these drugs may induce alterations in their normal intestinal flora, mainly through the acquisition of antibiotic-resistant and/or pathogenic bacteria [5], [6].

Even more critical is the situation of a number of insular populations of scavengers in the Macaronesian and Mediterranean archipelagos. Besides their high dependence on domestic livestock (wild prey populations have almost disappeared [8]), hunting, illegal poisoning, and the effects of pollutants have had a strong negative impact on individual survival [9]–[12]. As a result, several populations, some of them endemic, are at present severely endangered [9], [13], [14]. Within this framework, the characteristics inherent to insular populations (see below) could make insular scavengers especially vulnerable to the arrival of new pathogens mainly associated with the increasing mobility of livestock [15].

Pathogens are powerful selection agents, reducing individual fitness and thus able to drive rapid changes in population size, demographic structure, and the probability of persistence of their host populations [16]. The ecological and evolutionary differences between insular and continental scenarios may cause strong asymmetries in the exposition and susceptibility of vertebrates to pathogens. It has been suggested that insular populations have naturally impoverished pathogen communities [17], [18] and diminished immunocompetence, probably as a result of low exposition and reduced selection for parasite resistance during their evolutionary history [19]–[21]. Moreover, population constraints such as isolation, sedentary habits, high density and a reduction in genetic diversity make insular organisms especially susceptible to infection [22]–[25]. Consequently, pathogen exposure has been involved in the decline and even total extinction of vertebrates inhabiting insular systems [26]–[29]. This process may have become accelerated since growing human intrusion into wildlife habitat may have introduced new pathogens into such areas [5], [17], [22], [30].

The Egyptian vulture (*Neophron percnopterus*) is a medium-sized Old World scavenger considered to be ‘globally threatened’ whose world population has been recently estimated at 30,000–40,000 mature individuals. Migratory populations in continental Europe have suffered a decline of more than 50% over the last three generations and ongoing declines are occurring in other regions throughout the rest of its range [31]. Several sedentary insular populations still exist in the Macaronesian, Mediterranean, and Ethiopic archipelagos, making it an ideal model for testing whether insular vultures are more susceptible to the effects of the combination of factors outlined above. Taking advantage of parallel long-term studies in two areas of continental Spain and the Canary archipelago [32], [33], we compare here the vulture's vulnerability to pathogen infection and the impact pathogens have on individual health in two populations under two scenarios (insular *vs*. mainland) with socio-economic similarities (increasing intensification of livestock managing), but differing in ecological and biogeographical constraints (isolation, higher density, sedentarism and lower genetic variability of the insular population).

## Results

### (a) Pathogen survey

There was a general trend for pathogen prevalence (four of six taxa) to be higher in the insular population for both, fledglings and immature-adult birds. Prevalence of *Salmonella* spp. and *Candida albicans* was significantly higher in Canarian than Iberian fledglings (Table 1). The serological typing of Canarian birds showed a high prevalence of antibodies against *Salmonella enteritidis* (fledglings: 26.47%; immature-adults: 20%) and *Salmonella typhimurium* (fledglings: 26.47%; immature-adults: 25%) (Table 1). The bacteria *Mycobacterium avium* was only found in fledglings (6%) and immature-adults (10%) from the Canary Islands; the difference between regions was not significant, however, probably as a consequence of the small sample size. The prevalence of *Escherichia coli* O-86 was only examined in the insular population, being similar in fledglings (23.53%) and immature-adults (15%) (Fisher exact test, df = 1, *p* = 0.43).

**Table 1:** Prevalence and comparison of pathogen species in fledglings and immature-adults from the Iberian Peninsula and the Canary Islands.

	Fledglings			Immature/Adults		
Pathogen species	Iberia	Canary Islands	*p*	Iberia	Canary Islands	*p*
*Candida albicans*	0.38 (13/34)	0.68 (23/34)	**0.007**	0.36 (4/11)	0.55 (11/20)	ns
*Salmonella* (all serotypes)	0.06 (2/34)	0.32 (11/34)	**0.003**	0.09 (1/11)	0.30 (6/20)	ns
*Chlamydophila psittaci*	0.59 (20/34)	0.59 (20/34)	ns	0.50 (5/10)	0.45 (9/20)	ns
*Trichomonas gallinae*	0.56 (19/34)	0.71 (24/34)	ns	0.60 (6/10)	0.65 (13/20)	ns
*Mycobacterium avium* (culture and PCR)	0.00 (0/35)	0.06 (2/34)	ns	0.00 (0/10)	0.10 (2/20)	ns
*Mycoplasma* spp.	0.56 (19/34)	0.56 (19/34)	ns	0.40 (4/10)	0.40 (8/20)	ns

Significant differences are shown in bold; ns = not significant (*p*>0.008 after Bonferroni adjustment).

A clear association was found amongst pathogens in the Canarian population. The presence of *Chlamydophila* was associated with a higher prevalence of *Mycoplasma* in fledglings (*χ* ^2^ = 15.896, df = 1, *p*<0.001, contingency coefficient = 0.57, p<0.001) (Fig. 1) and with a higher prevalence of *Salmonella* (*χ* ^2^ = 5.09, df = 1, *p* = 0.024, contingency coefficient = 0.45, p<0.024) and *Mycoplasma* (*χ* ^2^ = 4.85, df = 1, *p* = 0.028, contingency coefficient = 0.44, p<0.028) in immature-adult birds. We did not find any type of associative patterns in the continental populations (*p*>0.05 in all cases).

**Figure 1:** Association between the pathogens *Chlamydophila psittaci* and *Mycoplasma* spp. in Canarian Egyptian vulture fledglings.

### (b) Individual immunocompetence

Multivariate tests for fledglings showed an overall significant effect of the Population (Wilks' λ = 0.36, F_11,29_ = 4.70, p<0.001, Partial Eta Squared = 0.64), the pathogens *Chlamydophila* (Wilks' λ = 0.34, F_11,29_ = 5.17, p<0.001, Partial Eta Squared = 0.66) and *Mycoplasma* (Wilks' λ = 0.41, F_11,29_ = 3.73, p = 0.002 Partial Eta Squared = 0.59) and the interaction between Population*Chlamydophila (Wilks' λ = 0.51, F_11,29_ = 2.53, p = 0.02, Partial Eta Squared = 0.49) and marginally between Population*Mycoplasma (Wilks' λ = 0.57, F_11,29_ = 1.97, p = 0.07, Partial Eta Squared = 0.43). Then, pair wise comparisons between estimated marginal means were done using Bonferroni adjustment for multiple comparisons. Canarian fledglings showed significantly lower levels of total white blood cells (F_1,39_ = 12.28, p = 0.001), heterophils (F_1,39_ = 10.29, p = 0.003), lymphocytes (F_1,39_ = 4.87, p = 0.03), monocytes (F_1,39_ = 24.19, p<0.001) and large lymphocytes (F_1,39_ = 5.84, p = 0.02). Moreover, Canarian fledglings infected by the pathogen *Chlamydophila* showed lower levels of lymphocytes (F = 4.80, df = 1, p = 0.034) and small lymphocytes (F = 4.51, df = 1, p = 0.040) and higher levels of basophiles (F = 4.40, df = 1, p = 0.042) than uninfected Canarian individuals. Multivariate tests for immature-adults birds did not show significant effects.

## Discussion

Insular Egyptian vultures had both a higher prevalence and frequency of association of avian pathogens and a poorer immune system. In addition to a reduced capacity for fighting pathogens, other factors such as the use of livestock and host density may explain the differences in pathogen incidence. Most of the reported pathogens are associated with intensively raised livestock [34], [35], [36] and so a higher prevalence of pathogens may be related to a greater reliance on these type of carcasses. However, carcass consumption is lower in insular Egyptian vultures (8% of prey items correspond to intensively raised livestock vs. 25.8% in the Ebro Valley [5]). Alternatively, high host density may increase pathogen spread and transmission efficiency [17]. On Fuerteventura Egyptian vultures come into contact with each other continuously throughout the year, not only at the “vulture restaurant”, but also at other feeding points (*corrals*) and communal roosts [9]. Mainland populations, on the contrary, are more segregated on their breeding grounds from both an intra- and inter-populational standpoint [37]. Unfortunately, because this species is becoming so rare, it is extremely difficult to test this possibility directly by comparing insular and continental Egyptian vulture populations of differing densities.

Within the Canary Island population we found a clear association between different pathogens in both fledglings and immature-adult birds. These associations usually appear when an opportunistic pathogen meets a host already weakened by a previous pathogenic infection [38], [39]. Interestingly, the Egyptian vultures in the Iberian Peninsula are exposed to the same pathogens (in fact, probably more exposed as they rely more on intensively farmed livestock), but no pair of pathogens was found to occur in one individual more or less often than chance would indicate.

These results suggest that Canarian vultures are more susceptible to infection by the same pathogens, which would imply that their immune response to them is weaker. Further evidence for this lies in the fact that, besides having higher rates of infection, Canarian fledglings showed lower leukocyte profiles for cells such as heterophils, lymphocytes, and monocytes that are crucial for an adequate innate and/or acquired immune response (see methods for the specific function of each cell type); when faced with infection these cells should circulate in proliferation [40], [41]. Moreover, Canarian fledglings infected by *Chlamydophila psittaci* showed lower rather than higher levels of lymphocytes and small lymphocytes (although they did have higher levels of basophils), which suggests that the immune response of these birds is inefficient and is not able to properly respond to infections [40], [41]. Finally, the idea that the Canarian population of Egyptian vultures is more susceptible to disease is reinforced by the presence in some birds of *Mycobacterium avium*, a ubiquitous pathogen generally affecting inmunocompromised animals [42], [43]. The lower immunocompetence is probably more noticeable in nestlings as their immune system is still developing [44]. Hence, the results of the necropsies and egg-content analyses performed (see methods) suggest that pathogens (mainly *Salmonella* spp., *E. coli* O-86 and *Chlamydophila psittaci*) play an important role in breeding failure in the Canarian Egyptian vulture population, which has the lowest known breeding success for this species within its distribution (0.5 fledglings/pair/year, [9]). Thus, disease-related mortality of fully grown fledglings in the nests is relatively high in Canary Islands (6.25% in 2002 N = 16), unlike in continental populations where almost no similar cases have been found in the 70 territories monitored annually (on average) in the Mid-Ebro Valley (1986–2005) [33] and the around 30 territories monitored annually in Cádiz (2000–2007) (authors unpublished).

Although no effects of pathogens were detected on the immune system of immature-adult vultures, the association found between *Chlamydophila psittaci*, *Mycoplasma* spp., and *Salmonella* spp. in Canarian birds suggests that the patterns found in fledglings may also exist in full-grown birds. Immature-adults may thus be ‘chronically-infected individuals’, that is, survivors that have developed acquired immunity after early infection by those pathogens. In fact, we found antibodies against *Salmonella* serotypes in immature-adults, indicating that these individuals had been exposed to this pathogen in the past. Alternatively, these individuals may be merely ‘tolerating’ the infection without eliciting an immune response. This may occur particularly under certain conditions such as stress, behavioural constraints (e.g. breeding), or the bioaccumulative effect of pollutants (heavy metals), which would prevent birds from assuming the high costs of an activated immune system [45]–[47]. In this sense, it should be noted that the sedentary habits of these vultures make them especially sensitive to lead intoxication originating from hunting activities [9], [12]. Lead interferes with the normal regulation of immune functions, leading to increased susceptibility to infection [48]–[50]. This poor immunocompetence may be mediated by the lower genetic variability found in Canarian Egyptian vultures [9], [51]; consequently, negative effects operating on the host's immune system may be expected to occur [25], [52], [53].

Given that we did not conduct any experiments on animals, our results are correlative but still compatible with a scenario of immune naïveté in insular vertebrates; their immune systems have evolved in an environment with a naturally impoverished pathogen community and are incapable of fighting efficiently against newly arrived pathogens [54]–[58]. Pathogen pressure is expected to influence the immune function since immune investment is a balance between costs and benefits, and investment is wasted in an environment without pathogens that need to be fought [59]. The arrival of new pathogens has been favoured by the increasing globalization and intensive management of livestock, which involves the frequent importation of animals to islands from the mainland [60]–[62]. In fact, the importation of sheep, pigs, and goats into the Canary Islands has dramatically increased in recent years (http://www.gobiernodecanarias.org/agricultura/otros/estadistica/default.htm). Consequently, island vultures are now probably more exposed than ever to potentially fatal multiple infections by pathogens typically acquired from livestock [34], [35], and to which they are supposedly naïve and thus far more susceptible [63].

### Implications for conservation

The scenario described in this study may occur in other insular Mediterranean and Macaronesian systems where populations of scavenger birds of prey are in serious decline and are gravely threatened [14], [32]. Livestock practices are powerful mechanisms of landscape engineering [8], [64], [65], but may also have major implications for the health of wild insular species [66]. The intensification of farming is occurring on a global scale and the disposal of carcasses of intensively raised livestock entails risks for scavengers [5], [6], [67], [68], which may be more serious for insular populations that have a weaker response to the arrival of novel pathogens with which they have had neither opportunity nor time to co-evolve [69], [70]. Not only scavengers but entire island bird communities are interlinked with traditional human activities sharing habitats, vectors, and pathogens with domestic species [66], [71]. Extreme caution should be thus taken when importing foreign livestock into insular systems in order to reduce the irruption of new pathogens into these especially naïve and fragile environments.

## Materials and Methods

Vulture monitoring was carried out on the island of Fuerteventura (Canary archipelago, 1662 km^2^) where there are 30 breeding pairs plus around 100 non-breeding birds [9] and in the Iberian Peninsula, where there is a widespread population of around 1,500 breeding pairs [72]. We chose two main continental study sites: the mid-Ebro Valley (northern Spain; 100 pairs plus around 200–300 non-breeding birds, 19,000 km^2^) and Cadiz (southern Spain; 30 pairs, 9.500 km^2^). The study areas have been well described elsewhere [9], [32], [33]. Island populations show higher densities than that found in continental regions. In Fuerteventura there are 9 birds/100 km^2^ whereas in the Iberian populations densities are below 2 birds/100 km^2^ (author's own data). In all these regions vultures regularly feed on carcasses of domestic livestock, both located randomly in the field and left in the so-called ‘vulture restaurants’, that is, artificial feeding stations where supplementary food for scavenger birds is provided [73] (authors' own data). The reliance on artificially supplied livestock carcasses is high for both populations. However, the rate of intensively raised livestock/wild preys in the diet of Egyptian vultures is greater in the Iberian Peninsula [5].

The capture and ringing of the birds was done under permits of the Spanish ‘Ministerio de Medio Ambiente’. Blood sampling and research protocols were authorized by the Regional Governments ‘Consejería de Medio Ambiente’ of Andalucía, Aragón, Navarra and Canarias.

### Sampling procedures

During 2004–2005 over 70 fledglings (36 continental and 34 insular) and 31 immature adults (11 continental and 20 insular) were captured at nest-sites or with cannon-nets. Blood samples (5 ml) were collected from the brachial vein. All the birds were handled following identical protocols and the time spent in collecting samples was almost identical for all individuals to avoid the possible among-individual variation in stress-induced alteration of the immune measurements.

### Pathogen survey

We conducted a comprehensive study of mycoplasmal, chlamydial, bacterial, fungal, and protozoan infections for a total of seven species: *Mycoplasma* spp., *Chlamydophila psittaci*, *Salmonella* spp., *Escherichia. coli* O-86 (enteropathogenic strain), *Mycobacterium avium*, *Candida albicans*, and *Trichomonas gallinae*. These pathogens are considered to be responsible for emerging infectious diseases [15], [49], [50] and were selected due to their known severe pathogenicity in birds. The effects of infection are variable, ranging from asymptomatic to severe disease with high mortality, as well as embryonic and neonatal mortality. Generally, transmission occurs by direct contact with infected individuals or through the consumption of contaminated food remains [43].

Some of them are primary pathogens, such as the enteric bacteria *Salmonella* spp., *Escherichia. coli* O-86 and *Chlamydophila psittaci*. The first two bacteria have caused disease in scavengers, such as colibacilosis in Red Kites (*Milvus milvus*), Cinereus vultures (*Aegypius monachus*) and Egyptian and Bearded vultures (*Gypaetus barbatus*) [5,6,74; author's unpublished). The list of avian species in which *Chlamydophila psittaci* infections occur is rapidly increasing. Wild avian species sharing aquatic or moist soil habitats with domestic poultry and granivorous birds may become infected via contaminated water and dust inhalation. The consumption of infected carcasses may transmit *C. psittaci* to host species that are predators or scavengers of other birds [75]. Host age can affect disease course after *C. psittaci* infection: adult birds may have asymptomatic infections, while young birds have acute disease [76], [77]. The others are mainly opportunistic pathogens, which generally infect immunodepressed individuals or those individuals first affected by a primary pathogen. At present, this is the main way of pathogen acquisition in scavenging birds in Spain [68]. For example, the widespread pathogen *Candida albicans* is found in very high prevalence in Black and Griffon vultures (*Gyps fulvus*) causing severe disease, especially in immunocompromised individuals [6].

0Most of these pathogens are present in intensively raised livestock [68], [78]. Moreover, *Salmonella* spp., *Escherichia coli* O-86 and *Candida albicans* are saprophytic bacteria normally associated to the accumulation and decomposition of livestock carcasses at vulture's restaurants. *Mycobacterium avium* is generally associated to extensive livestock from where it can be acquired by scavenger birds [79]. A recent *Mycobacterium bovis* and serotype VII *M. avium* outbreak is causing disease and mortality in nestlings and juveniles of Griffon vulture populations in central Spain (authors, unpublished data).

As a previous work, after the verification of breeding failure, we developed the analyses of egg content (three unfertile eggs and four embryos) and necropsy of two dead fledglings from Canary Islands. It revealed the presence of several pathogens compatible with fatal septicaemia in eight birds: the commonest pathogens were *Salmonella* spp., *E. coli O-86*, and *Chlamydophila psittaci*, while *Erysipelothrix rhusiopathiae* was isolated from the corpse of one of the fledglings (authors unpublished).

### Microbiological isolation

Bacterial microflora was sampled from the cloaca, choana, and nares of individuals with sterile microbiological swabs and Amies transport medium. Samples were transported in a cool container to the laboratory within 12 hours of collection and were processed within one to two hours of arrival.

For *Salmonella*, microbiological methods were used for cultivation and isolation, and for serotype identification, as described elsewhere [74]. Serology for *Salmonella* spp. was performed when no cloacal samples were taken. In this case only *Salmonella typhimurium* and *Salmonella enteritidis* antisera were used, because they are the most common serotypes isolated from raptors [80]. Serological tests are satisfactory for establishing the presence and estimating the prevalence of infections [35], [80]–[82]. This rapid whole blood-plate agglutination test used the antigen Difco (TM) *Salmonella* O Group B Antigen (1–4–5–12) (Becton Dickinson and Company, Maryland, USA). The test was conducted by using the manufacturer's standard instructions [83]. For the determination of *Mycobacterium avium*, cloacal and tracheal samples taken with sterile swabs were plated on Lowenstein-Jenssen media and incubated for three months. Samples with *Mycobacterium* growth were stained (Ziehl-Nielsen and auramine rhodamine acid-fast stains) and PCR techniques were used to identify the agent. These techniques have been proved to be adequate for the isolation of this pathogen in wild fauna [84], [85]. The presence of the *Mycobacterium* was considered to be proven when both cultures and molecular techniques were consistent [86]. Clinical *Candida albicans* was determined by the examination and sampling of oral cavities. Samples were cultured in standard fungical media (Agar Sabouraud) at 37°C for 48 hours. The presence of *Escherichia coli* O86 (enteropathogenic strain) was determined by phenotypic and genotypic characterization [87] and by PCR [88]. *Mycoplasma* spp. and *Chlamydophila psittaci* were determined by PCR. For the determination of strains we followed the protocols published by [89]. *Trichomonas gallinae* was determined by direct visualization in warm physiologic solution, culture [90] and PCR [91].

### Immune assays

We evaluated individual immunocompetence by measuring several cellular and humoral immune system parameters. After blood samples collection, approximately 4 ml was transferred to a lithium-heparinized tube and immediately refrigerated at 4–6°C. In addition, two blood smears were obtained immediately for each individual and fixed for three minutes with methanol and stained with May-Grünwald Giemsa stains for haematological parameter determination. Details of the haematological techniques and parameters were standard and can be found elsewhere [40], [92], [93].

Leukocyte concentrations provide information on circulating immune cells which can be used as an indicator of health [40]. The immunological function of each of the white blood cells (WBC) types has been reviewed extensively elsewhere [41], [94], [95]. Briefly, heterophils are the primary phagocytic leukocyte and mediate innate immunity against novel pathogens. Lymphocytes are involved in several immunological functions, such as immunoglobulin production and modulation of immune defence [40]. Eosinophils and basophils play a role in the inflammation process [40], [94] and the first are associated with defence against parasites [96]. Finally, monocytes are long lived phagocytic cells associated with defence against infections and bacteria [40].

The total WBC count was determined by counting all leucocytes in a Neubauer chamber and multiplying the raw data by 200 to obtain the final values [40]. The proportion of different types of leucocytes was assessed on the basis of an examination of a total of 100 leucocytes under oil immersion. Plasma was separated by centrifugation at 3,000 r.p.m. for 10 minutes within eight hours of extraction and then stored at −20°C. Plasma samples were used for protein plasma electrophoresis and serology tests (immunoglobulins: α, β and γ –globulins) [97].

### Statistical analyses

#### (i) Prevalence

The prevalence of six pathogen species (number of infected individuals/number of sampled individuals) in insular and continental populations was compared using contingency tables (χ^2^ test), which accounts for the nature of the prevalence data (frequencies) and the unbalanced sample sizes [98]. The bacterium *E. coli* O-86 (enteropathogenic strain) was examined only in the insular population.

As a previous step, we compared the prevalence between the two continental populations. We found no differences (*p*>0.05 in all cases) and so the data from the two continental populations were pooled (hereafter Iberia). We kept the data pool separated in age groups because it is well known that the immune system of adult birds differs from that of fledglings since the later need some time to mature and be efficient [99]. Since multiple tests were carried out we adjusted the α-level using the Bonferroni correction for each data set (fledglings and immature-adults). The association between pathogen species was analyzed by means of contingency tables (χ^2^ test) controlling for the variable “population” and measured by means of contingency coefficients.

#### (ii) Effect of pathogens

To determine whether the effect of pathogens on the immune response differed between populations we used multivariate analyses of variance MANOVA, which allow an overall test of the effects of the explanatory variables evaluating cellular and humoral immune response (differential counts of WBC: total WBC, heterophils, lymphocytes, large lymphocytes, small lymphocytes, monocytes, eosinophils and immunoglobulins: α, β and γ –globulins). In order to avoid inherent variance to different immune response between fledglings and immature-adult individuals [97], we carried out separate factorial-MANOVA analyses for each age class (sum of squares type III). When normality was not attained (Shapiro-Wilk tests), variables were transformed accordingly. The Levene contrast was applied in order to test the equality of the error variances for each response variable (p>0.05 in all cases). Population (1 = continental or 2 = insular) and six pathogen species were included as factors in each analysis. Whenever the sample size was appropriate, we considered the interactions between the population and each pathogen species. Moreover, we controlled for the possible effect of the remaining variables evaluating immune system and body condition (mean corpuscular volume MCV, mean corpuscular haemoglobin MCH, and mean corpuscular haemoglobin concentration MCHC) and included them as covariates in the model.
